The article "Optimization of Tennis Teaching Resources and Data Visualization Based on Support Vector Machine" was published in 2022. Journal: Comput Intell Neurosci.

# Optimization of Tennis Teaching Resources and Data Visualization Based on Support Vector Machine

**DOI:** 10.1155/2022/4672586

**Published:** 2022-08-29

**Authors:** Shaokun Zhang, Huan Yu

**Affiliations:** ^1^Physical Education Institute, East China Jiaotong University, Nanchang, Jiangxi 330000, China; ^2^Physical Education Institute, Shangrao Normal University, Shangrao, Jiangxi 334000, China

## Abstract

In recent years, with the continuous development of machine learning technology, this technology has achieved success in many fields and activities. Therefore, using machine learning technology for fuzzy research has a good research prospect. In the development of related research, the author of this study noticed that some researchers began to use tennis machine learning technology and achieved good results. However, most of the research is only for simple analysis and is related to the current work. It cannot be used to move a solid tennis ball, nor it can make small changes to the original tennis movement; thus, it cannot carry out a complete and brand-new movement. The defense of tennis first establishes visual teaching tools with the help of various courses and visual teaching techniques to improve the teaching effect. By optimizing the network data, this study constructs the corresponding data search model, which downloads a large amount of data from the network ram, so as to separate the impact of the network environment on the load. The simulation results show that the model is optimized for the high-quality 3G network environment, and the load time and energy consumption are greatly reduced. It is more efficient in WiFi and a a high-quality 4G network environment.

## 1. Introduction

The current solution for “power-based optimization” for mobile network applications is power consumption analysis, where energy needs to be measured, analyzed, and adjusted, as well as such things as network connection status, user experience, consumer behavior, local network, and information [1]. The dense environment will affect the energy consumption in mobile network applications. This article focuses on the use of energy and performance management plans, these plans are related to the import of mobile network data and mobile web browsers, using the most appropriate method to reduce Lyapunov, support vector machine algorithm format [2]. In recent years, with the rapid development of computer and Internet technology, human society has entered a period of information explosion, and people have to deal with a large amount of information every day [3]. Consumer needs continue from data acquisition and access to effective and cost-effective information development. Considering the origin of the times, the continuous development of information retrieval technology is also a priority for emerging technologies [4]. The combination of machine learning and teaching visualization inevitably becomes a model, and the method of combining the two is used in tennis [5]. Fictional teaching is a theory, method, and technology that uses computer graphics and visual processing technology to convert data into shapes or images, and then displays them on the screen, and then based on advanced educational design concepts, supported in a multidisciplinary technical environment. Then, based on the advanced educational design concept, it carries out the next step of interaction in the multidisciplinary technology environment [6]. The course is rich in resources, reasonable in structure, and open to the environment. It can develop students' independent learning and innovative thinking abilities, and help teachers and students communicate and learn effectively [7]. According to the tenet of tennis teaching, we have chosen a variety of learning methods, such as watching teaching videos, enhancing memory, effective practice, case analysis, video feedback, training, thinking, etc., and we have also improved the integration and designed it as a daily goal for teaching [8]. The basis for the modification of traditional teaching methods and visual teaching methods. The defense of tennis first uses various courses and visual teaching techniques to establish visual teaching tools to learn visual targets for teaching goals, teaching methods and feedback loops, thereby improving the teaching effect [9]. The principles of tennis defense and visual learning use a variety of media to stimulate students' interest in learning, help students quickly establish technical representations of sports, learn correct sports thoughts, and improve intelligence and the use of technical tools [10]. Improve students' thinking skills and better understand the nature of strategies.

## 2. Related Work

The literature introduces the comparison of infrared target imaging and recognition technology: if the target itself is small, or the distance between the target and the non-imaging system is too far, the imaging area of the target is small, and only visible points or point vision, infrared target detection is more complicated [11]. The literature introduces the classification and recognition of surface infrared technology based on vector machines: the image area of surface targets is much larger than the target infrared imaging system, and the same person wearing different clothes has different characteristics to be observed [12]. The literature introduces that SVM + HOG supports a classification [13]. The method is to add the GLCM algorithm to capture the appearance and shape of the target, classify and identify the infrared target above, and solve the problem of changing infrared radiation target recognition in different clothing [14]. The literature introduces the research of infrared flying target and ground pedestrian detection based on neural convolutional network: infrared target detection and ground pedestrian detection. Two ideas are adopted to solve this problem. The literature introduces the data collection, defines the development process and research status of search and classification algorithms, defines the structure of the classification learning process, and provides guidelines for classification and analysis, research, and improvement of the following algorithms.

## 3. Mobile Network Power Consumption and Dynamic Optimization Machine Learning Model

### 3.1. Optimized Architecture Design of Fuzz Testing Resources Based on Machine Learning

Due to the inefficiency of existing fuzzing methods and the lack of code (especially hard copy files such as PDF files), there is no solution to create a brand new file in the process of creating a new PDF to improve the quality. To this end, this study proposes a learning structure based on seed files, as shown in Figure 1. This structure studies the grammar and relationship between the seed file and the original seed through a machine learning process, so as to obtain the form of genetic speech. Then, we used this extraction method to identify new files to create PDF, and finally, we used a new generation of AFL fuzzer tool to study the improvement of the guaranteed rate.

Our entire structure can be divided into three parts: the first part is the structure of the PDF objects that make up the corpus; the second part is the structure of the PDF objects that make up the main body; the third part is the PDF file wrapper.

The Markov chain structure is a streamlined process, describing one area as another area. Specifically, if the probability of regional transition is met, a series of regions *X* = {*X*_1_, *X*_2_, *X*_3_}:

(1) $$\begin{array}{c} p\left(X_{t+1}|X_{t},\ldots ,X_{1}\right)=p\left(X_{t+1}|X_{t}\right). \end{array}$$

The encoder operates in the order of insertion. After a series of length conversions by the encoder, a medium-length vector *c* is obtained. The calculation method of *c* is shown in formula (2):

(2) $$\begin{array}{c} c=q\left(h_{1},h_{2},\ldots ,h_{n}\right). \end{array}$$

Along with the following equation:

(3) $$\begin{array}{c} h_{i}=f\left(x_{t},h_{t-1}\right). \end{array}$$

After the hidden layer variable, the hidden layer at time *t* is then:

(4) $$\begin{array}{c} h_{t}^{\prime }=g\left(y_{t-1},c_{t},s_{t-1}\right). \end{array}$$

Sequential networks usually use different types of repetitive neural networks as the main unit, the most commonly used is the long-term memory network (LSTM). The short storage network, called the LSTM network, is an RNN-like network. Since the RNN network is trained, the creation of the next node is related to the information of the previous node, so if the sequence is too long, it is easy to cause surface loss. The function expression is represented by formula (5):

(5) $$\begin{array}{c} S\left(x\right)=\frac{1}{1+e^{-x}}. \end{array}$$

It can be seen from the Sigmoid display that the value of *S*(*x*) is between 0 and 1. After conversion, the classification *S*(*x*) can be used to find:

(6) $$\begin{array}{c} S\prime \left(x\right)=\frac{e^{-x}}{{\left(1+e^{-x}\right)}^{2}}=S\left(x\right)\left(1-S\left(x\right)\right). \end{array}$$

The forget gate is the most important part of the short storage network LSTM, it knows the available information and forgets the information. In principle, it is expressed by formula (7):

(7) $$\begin{array}{c} f_{t}=\sigma \left(W_{f}\left[h_{t-1},x_{t}\right]+b_{f}\right). \end{array}$$

The update gateway is used to determine what information will be included in the LSTM network segment. It consists of two parts: an entrance door made of S-shaped activities and a generator made of tanh activities. The performance of tanh activity is represented by Equation (8):

(8) $$\begin{array}{c} \text{tan}h\left(x\right)=\frac{e^{x}-e^{-x}}{e^{x}+e^{-x}}. \end{array}$$

Since the introduction and extraction of tanh(*x*) can continue in an indirect and monotonous manner, there is no problem of vanishing gradients. Therefore, the principle of change is expressed by equations (9) and (10):

(9) $$\begin{array}{c} i_{t}=\sigma \left(W_{i}\left[h_{t-1},x_{t}\right]+b_{i}\right), \end{array}$$

(10) $$\begin{array}{c} {\tilde{C}}_{t}=\text{tan}h\left(W_{C}\left[h_{t-1},x_{t}\right]+b_{C}\right). \end{array}$$

For update gates and forget gates, the input is determined by formula (11):

(11) $$\begin{array}{c} C_{t}=f_{t}*C_{t-1}+i_{t}*{\tilde{C}}_{t}. \end{array}$$

The last gate is the output gate, which determines the content of the output. As shown in Equations (12) and (13), the production gateway is divided into two steps that operate in the unit state, and the final output of the production gateway is the product of the results obtained by the two manufacturing functions.

(12) $$\begin{array}{c} o_{t}=\sigma \left(W_{o}\left[h_{t-1},x_{t}\right]+b_{o}\right), \end{array}$$

(13) $$\begin{array}{c} h_{t}=o_{t}*\text{tan}h\left(C_{t}\right). \end{array}$$

### 3.2. Simulation Experiment Results and Analysis of Mobile Network Power Consumption Combination Algorithm

Network delay refers to the time required to transmit data packets across the network, especially the time from the head of the data packet entering the input port to the end of the data packet leaving the output port. Network delay usually consists of two parts, one is the delay, in this case, looga needs to transmit the packet data to the network time, and the other is the serial delay, that is, the time required to pack the data. Its expression is represented by formula (14).

(14) $$\begin{array}{c} L\left(\text{cycles }\right)=T_{\hbar }+T_{s}, \end{array}$$

*L* represents the delay of data packets, so the total network delay must be the total delay of all data packets divided by the total number of data packets. According to formula (15).

(15) $$\begin{array}{c} \bar{L}\left(\text{cycles}\right)=\frac{\sum_{i=1}^{N}Li}{N}. \end{array}$$

The network output size refers to the number of microchips available for each network node on a port per hour. Its expression is represented by formula (16).

(16) $$\begin{array}{c} T\left(\text{flit}/\text{Cycle}/\text{IP}\right)=\frac{\sum_{i=1}^{n}L_{i}}{N\times t}. \end{array}$$

The electrical power of the pipeline refers to the flow path used in the process of transmitting, storing, and processing data packets. Electricity in the corridor always includes electricity for storage and electricity for intersections. The literature describes the energy consumption of the pipeline in detail, and the mathematical formula is shown in formula (17).

(17) $$\begin{array}{c} P_{\text{router}}=E_{\text{router}}\cdot f_{\text{clk}}=\left(E_{\text{buffer}}+E_{\text{arbiter}}+E_{\text{Crossbar}}\right)\cdot f_{\text{clk}}. \end{array}$$

Due to the storage of the first production plan (FIFO), and repeated read and write operations, a lot of energy was wasted. Factors such as the number of virtual channels, FIFO depth, and FIFO data creation will affect input energy consumption. The formula for using energy storage is shown in formula (18):

(18) $$\begin{array}{c} E_{\text{buffer}}=n\cdot \text{depth}\cdot \alpha_{F}\cdot k_{1}. \end{array}$$

Crossbar switch is another component of node energy consumption. Yang Zhongming and others proposed a formula for calculating the energy consumption of cross-nodes, as shown in formula (19):

(19) $$\begin{array}{c} E_{\text{Crossbar}}=c_{1}\alpha_{c}+k_{3}. \end{array}$$

The ability to use a communication link refers to the power lost in the transmission path during the transmission of data packets from one node to another network. As the level of nano-production technology is gradually introduced, the line width continues to decrease, and the consumption of power communication media increases with the ability to operate the entire system. If the power consumption of network communication can be effectively reduced, the overall power consumption of the bottom layer will also be reduced. Therefore, how to reduce the energy consumption of the communication network has always been the focus of research on the energy consumption of the network on a chip. Kahng et al. proposed a formula for using electricity in the calculation (20) and a formula for communication (21).

(20) $$\begin{array}{c} P_{\text{link}}=\alpha \cdot C_{l}\cdot v_{d\;d}^{2}\cdot f_{\text{clk}}, \end{array}$$

(21) $$\begin{array}{c} C_{1}=C_{in}+C_{\text{gnd }}+C_{CC}. \end{array}$$

The operating system environment used in this experiment is Linux, and the emulator used is Noxim. The parameter structure required for the test is shown in Table 1. This article chooses 2D-Mesh as the on-chip network architecture mainly because it is compatible with the router-based design of the general architecture and is often used for network testing. In order to verify the blockchain function of the algorithm in this study, four virtual channels are used for network connection. The routing algorithm used in this article is the XY algorithm because XY is a standard decision-making method and is usually used as a reference method. In order to ensure the accuracy of the experiment, this article uses 2000 cycles to ensure that the data related to the experiment is not included in the analysis of the experimental data, so that the simulation data can be collected correctly. The aggregation algorithm in this article compares the XY algorithm, NoP algorithm, and CRA algorithm for different traffic patterns.

The main run_simulation diagram shown above is shown in Figure 2. Usually need to run the entire computer, the ultimate goal is to obtain the necessary information in this article. The standard overall structure of the network chip and network adapts to many operations of looga in this article, the rules of production, delay, and power consumption data components.

This section describes the use of network power for any random integrated transpose 1 and transpose 2 formats. In nothing else, if the injection rate is greater than 0.015, the difference in power consumption between the various algorithms begins to become obvious. The utilization rate of the Hybrid algorithm is 13% lower than that of the NoP algorithm and 10.5% lower than that of the NoP algorithm. In the conversion method, if the pointer threshold is greater than 0.02, the difference in power consumption between several algorithms will begin to be visible. The utilization rate of Hybrid algorithm is 11.2% lower than that of the NoP algorithm and 8.5% lower than that of the CRA algorithm. In Transpose 1 and Transpose 2, if the size of the needle is greater than 0.015, the difference in power consumption between several algorithms will begin to be visible. In transpose 1, the power consumption of the Hybrid algorithm is 11.7% lower than that of the NoP algorithm and 10.6% lower than that of the CRA algorithm. In the transpose 2 model, the power consumption of the Hybrid algorithm is 12.4% lower than that of the NoP algorithm and 10.1% lower than the power consumption of the CRA algorithm. Compare the simulation results in this study with the design indicators at the top and bottom of the NoP algorithm and the CRA algorithm. The power consumption reduction of the CRA algorithm is very small, and the function of the path summation algorithm is not as powerful as the NoP algorithm and the CRA algorithm. Through the comparison and analysis of the simulation results and the design indicators, it is found that the simulation results in this study have reached the first design indicators, as shown in Table 2.

### 3.3. The Performance and Power Consumption Optimization Strategy of Mobile Network Applications

Apply the MDP model built into the first part of the Android live music device and notify it directly when downloading a new import application. During the trial period, 10 users submitted download requests at any time within two hours. EDM will check the MDP judgment table according to the current time, volume, signal strength, and queue length, and finally decide the action to be taken (import/delay). In order to complete the analysis of the EDM performance shown in this unit, we compared the LM import strategy with the powerful LM and Android system import strategy. LLA decided to respond to the import task by following Lyapunov's repair procedures and optimizing the customer model, and it is better to choose wireless access to complete the data transmission. This method selects powerful connections to complete the import task by analyzing the local data of the mobile device and the current state of the network. The core of LLA is the unit W, which affects input energy consumption and time delay. A small amount of W can reduce the delay time, but it will increase the download power consumption. A large amount of W will reduce energy consumption, but will lead to negative use. Allow *W* = 22. This test allows 10 users to copy import requests within two hours according to different usage conditions (light use *p*=0.2, average use *p*=0.5, heavy use *p*=0.8), education level and minimum delay EDM use of the three strategies and capabilities to utilize average energy, energy efficiency, and latency. *E* represents the average energy consumption per person, *D* represents the average delay time per person, *T* (IC … *N*_req1_) represents the time used in the settlement process *i*, and *D* (*i*…*N*_req_) the delayed work response time *i*. In addition, the performance index is defined to evaluate the energy efficiency of various import strategies.

(22) $$\begin{array}{c} \bar{E}=\frac{\sum_{i=1}^{N}T\left(i\right)\times \text{Power}}{\text{FileSize }N},\\ \bar{D}=\frac{\sum_{i=1}^{N}D\left(i\right)}{\text{FileSize }xN},\\ \text{Performance}=\bar{E}\times \bar{D}. \end{array}$$

This section uses the example tree decision method, uses SVM and tree creation algorithm to build a more appropriate strength structure modeling model, and compares the variance estimates of the two variables. First, use the *R*_part_*r* software package to analyze 400 website functions and classification functions, and directly create a tree, and the other 100 pages are used for experimental samples. Experimental results show that the classification accuracy rate is only 42.7%. In order to avoid excessive logging issues, a review tree was also designed, reducing production time by 39%. SVM is a global classification algorithm that regularly uses all symbols to construct non-overlapping parts. Since the functions in this unit are small and the training scale is small, the RBF radio function is selected as the SVM kernel task. The penalty factor *C* and the width of the kernel function are two important determinants that affect the accuracy of SVM-RBF classification. *C* defines the amount of error data, which is a special unit called RBF. If the value C is too short, a classification result with short deviation and high variance will be produced, and if the value *C* is too large, there may be a classification result with high deviation and small variance. This machine uses e1071 in the R software package to create an SVM model, and uses the built-in SVM. Tune function (a web search method) to find the maximum value and classification of *C*. Experiments show that under the maximum intensity, the variability of the accuracy of the prediction model can reach 88.9% (*C* = 100, *y* = 0.01). The function of the SVM prediction model is shown in Figure 3.

This model downloads a large amount of data from the network RAM, thereby separating the influence of the network environment on the load. This section considers the same energy consumption and load parameters and studies the loading conditions of web pages on devices under different quality environments.

This section discusses how to predict model examples in real network environments. Use virtual networks to match 2G, 3G, 4G, and WiFi networks. The detailed boundary is shown in Table 3. Each network environment is divided into two parts: a high-quality network communication environment and a poor-quality network communication environment (if the packet loss rate is higher than 15%, it is worse). Odroid XU3 connects to the web page through a local server to test the network performance on different networks.

## 4. Application of Visualization Technology in Tennis Teaching Analysis and Countermeasures

### 4.1. Searching and Sorting Algorithm for Tennis Teaching Data Based on Machine Learning

ERR (reciprocal average ranking) refers to the expected ranking, which represents the expectation of meeting the user's requirements, rather than returning the most suitable position in the document calculated in the RR. The preliminary evaluation criteria considered site value information and related site document information but did not consider the relationship between documents. The public file has an important relationship with the previous file and is related to the previous file. If the ranking is short, the possibility of clicking this document is high. If the previous document is relevant, it is unlikely to push this document. In the application, I will no longer view other Use Go documents to indicate that the user may not be able to see other documents after viewing the current location. Therefore, the probability of a user at position *r* is as follows:

(23) $$\begin{array}{c} P_{r}=\prod_{i=1}^{r-1}\left(1-R_{i}\right)R. \end{array}$$

In addition, Ro is a document-related level function, you can choose the following options:

(24) $$\begin{array}{c} R_{i}=R\left(g_{i}\right)=\frac{2^{g}-1}{2^{g_{\text{max}}}},\;g\in \left\{0,1,\ldots ,g_{\text{max}}\right\}. \end{array}$$

The following ERR calculation formula is as follows:

(25) $$\begin{array}{c} \text{ERR}=\sum_{r=1}^{n}\varphi \left(r\right)P_{r}=\sum_{r=1}^{n}\frac{1}{r}P_{r}=\sum_{r=1}^{n}\frac{1}{r}\prod_{i=1}^{r-1}\left(1-R_{i}\right)R. \end{array}$$

The neural network adjusts the weight of the entire neural network by continuously amplifying backscatter, and finally reaches the initial frequency, or if the sample is known to reach a very good level, it will stop repeating. After the task is completed, train the neural network system.  Figure 4 is a schematic diagram of neural network path dispersion.

Ranking learning is a machine learning method, which means that the algorithm determines the function of the given training data (resistance model), and when new training data arrives, it can provide us with predictable results based on this work. This unit uses LETOR data, which is mainly used to obtain and classify conditional equipment. LETOR data was downloaded from Microsoft Research Asia, LETOR 1.0 version was released in April 2007, LETOR 2.0 version was released in July 2007, LETOR 3.0 version was released in December 2008, and LETOR 4.0.0 version was released in 2009, Released in July. The LETOR 4.0 version is very different from the previous version. LETOR 2.0 is an update of LETOR 1.0, while LETOR 3.0 is an update of LETOR 2.0, but LETOR 4.0 is the new data for this version, which is available in MQ2007 and MQ2008 Two independent questions. Each question has related documents. The relevance of each question is marked at three levels (2, 1, 0), which means that we are very applicable, partially applicable, and not applicable. Each document creates 46 attributes based on documents, links, etc., and 46 different documents can be divided into about 9 categories, as shown in Table 4:

There are about 1700 application requests in MQ2007 and about 800 data requests in MQ2008. During the experiment, a cross-validation technique was used to divide the data into *S*1, *S*2, *S*3, *S*4, and *S*5 parts, and then group the data at 5 high places. Five categories according to different combinations, namely Fold 1, Fold 2, Fold 3, Fold 4 and Fold 5. Each section contains three subdivisions. Both MQ2008 and MQ2007 have 5 functions. Each data fold in MQ2008 contains a maximum of 2000 documents, and each data fold in MQ2007 contains a maximum of 9000 documents, as shown in Table 5.

### 4.2. Visual Analysis of the Quantitative Characteristics and Growth Law of Tennis Scientific Research Literature

The values believe that the development of literature can be divided into four cycles: slow growth and development, rapid growth, maturity and strength, and slow decline, decline, and extinction. The changes in the number of publications in recent years may better reflect the dynamics and basic developments in the field of research. Through extensive analysis of basic tennis journals in recent years, changes in development can be found. Tennis journals and the current development cycle paved the way for further research on tennis research literature and key concepts and foundations. The annual publication status refers to the collection of scientific literature in all journals of a specific category at a specific time of the year, and it is an indicator that reflects the changes in research on the subject. Find and download articles published in major tennis journals for many years through CNKI, and then classify, download, and count them, as shown in Table 6.

It can be seen from Figure 5 that from 1992 to 2005, the publication of Chinese Tennis Magazine was a period of slow and long-term growth. After 14 years of development, there is still some imbalance. This is the introduction of tennis in schools and the entire country. The development of tennis is still in its infancy, and the development of tennis is not very advanced. Local scholars do not pay attention to tennis. It has little impact on world-leading sports such as table tennis and basketball. As a result, unstable items have experienced rapid growth from 2006 to 2015. The growth rate is rapidly accelerating and changing The table shows a broad trend, indicating that at this time tennis research has attracted widespread attention, and the most productive situation is emerging. It can be seen from Figure 5 and Table 6 that during the period of slow growth, at least 56 articles were published in 2008, and the most published in 2015 was 207 articles, a slight decrease from 2009 to 2013. During the period of rapid growth, the number of articles published increased rapidly from 237 to 766 in 10 years. In the past two years, maturity and strength have been declining sharply. After analyzing the data at a high level, the change equation is: *Y* = 31.051*X* − 86.572, *R*2 = 0.8314. Among them, *R*2 is the determinant of the balance formula, which represents the reliability of the installed model, and when it is close to 1, it is the high reliability of the variable frequency map. In this formula, *R*2 is 0.8314, which can show an 83.14% consistency in the annual publication, and its reliability is very high. It can be seen from the relevant formulas and graphical changes that from 2009 to 2020, the number of tennis examination papers in China has generally shown a gradual increase.

In citation analysis, the number of conversations is an important unit and basic method of analysis. The number of citations refers to the number of other references cited in the literature, reflecting the background of material exchange and use of the literature. By analyzing the value of the citations on each topic, we can better understand the development of the material and the use of the researchers' literary works. The use of multiple references is influenced by many aspects, such as the author's writing skills. Overall, it is directly proportional to the author's ability to perceive and borrow information. Use advanced methods to classify and analyze the citation data of tennis research literature (Table 7). It can be seen from the table that among the 508 tennis articles, there are 447 articles with references, accounting for 88% of the papers. From 1992 to 2017, the citation ratio and the total number of documents were equivalent to 88% of domestic scientific journals, but lower than the average of 90% of foreign technical journals. However, the three themes of sports training, competition, and tennis learning are higher than the content of domestic and foreign journals. This shows that China's various disciplines are unbalanced in absorbing and utilizing the progress of literature. However, among the 508 census documents from 1996 to 2020, there are always 12,603 citations, of which 24.8 and 28.2 are citations, the highest being 8.86 citations in Chinese scientific journals, scientific and foreign scientific journals. Each journal article has been cited more than 15 times. It perfectly shows that, both domestically and externally, China's absorption and use of scientific research literature are above average.

## 5. Conclusion

From the invention and improvement of this study, the widespread use of printing to the emergence and rapid development of the Internet, the methods and speed of information transmission have changed. The amount of information is also increasing rapidly, enough to easily understand the latest tools and information today. This article starts with the research on classification algorithms and introduces the development background and current research level of classification algorithms, including the initial statistical classification of word frequency and word position, and then the hyperlink classification algorithm. It briefly introduces the three classification algorithms (pair-by-pair, point-by-point, and smart list) tailored for the next-generation search engine, their characteristics, and the analysis indicators of the performance algorithm. Next, conduct an in-depth analysis of the BP neural network structure, and analyze the specific operating mechanism of the algorithm. The structure studies the syntax and relationship between the seed file and the original seed through the machine learning process, so as to obtain the form of genetic speech. Then, we use this extraction method to identify new files to create PDF. Finally, we use a new generation of AFL fuzzer tool to study the improvement of the assurance rate.

## Figures and Tables

**Figure 1:** Fuzzing test framework diagram based on machine learning.

**Figure 2:** Run_simulation flow chart.

**Figure 3:** Configure SVM classification line and processor plan diagram.

**Figure 4:** Neural network backpropagation flowchart.

**Figure 5:** The development trend chart of the total number of tennis periodicals.

**Table 1:** On-chip network experiment configuration.

Parameter	Size
Network size	4*∗*4
Topology	3D-mesh
Virtual channel	4
Cache	4
Flit size	8
Flow pattern	Random, shuffle, transposal, transpose?
Deterministic routing algorithm	XY
Adaptive routing algorithm	NOP
Simulation cycle	100000 cycles
Initialization cycle	4000 cycles

**Table 2:** Comparison of design indicators and simulation results.

	Average delay		Throughput rate		Power consumption	
	Design specifications	Simulation results	Design specifications	Simulation results	Design specifications	Simulation results
NOP	Up to 6% increase	Increase 3.4%–4.0%	Up to 3% reduction	Decrease 2.6%–3%	At least 9% reduction	Decrease 11.1%–12%
CRA	Up to 8% increase	Increase 4.10%–4.8%	Up to 4% reduction	Decrease 3.2%–4%	At least 7% reduction	Decrease 8.4%–10.5%

**Table 3:** Different network environment parameters.

	Upstream	Down	RTT	Packet loss rate
2G excellent	50 Kbit/s	50 Kbit/s	200 ms	0
2G difference	50 Kbit/s	50 Kbit/s	200 ms	15%
3G excellent	2 Mbit/s	5 Mbit/s	5 Oras	0
3G difference	2 Mbit/s	5 Mbit/s	50 ms	15%
4G excellent	5 Mbit/s	10 Mbit/s	20 ms	0
4G difference	5 Mbit/s	10 Mbit/s	20 ms	15%
WiFi excellent	50 Mbit/s	50 Mbit/s	20 ms	0
Poor WiFi	50 Mbit/s	50 Mbit/s	20 ms	15%

**Table 4:** Features extracted from documents.

TF	TF of body	TF of anchor	TF of title	TF of URL	TF of whole doc
IDF	IDF of body	IDF of anchor	IDF of title	IDF of URL	IDF of whole doc
TF*∗*IDT	TF*∗*IDT of body	TF*∗*IDT of anchor	TF*∗*IDT of title	TF*∗*IDT of URL	TF*∗*IDT of whole doc
DL	DL of body	DL of anchor	DL of title	DL of URL	DL of whole doc
BM25	BM20 of body	BM20 of anchor	BM20 of title	BM20 of URL	BM20 of whole doc

**Table 5:** Cross-validation data set partition.

Folds	Training set	Validation set	Test set
Fold l	{*S*1, *S*2, *S*4}	*S*4	*S*2
Fold 2	{*S*2, *S*3, *S*5)	*S*5	*S*3
Fold 3	{*S*2, *S*4, *S*5)	*S*1	*S*5
Fold 4	{*S*1, *S*4, *S*5)	*S*2	*S*4
Fold 5	{*S*1, *S*3, *S*5)	*S*3	*S*1

**Table 6:** Basic status of tennis research literature.

Year	Core volume	Cumulative amount	Total	Percentage	Year	Core volume	Cumulative amount	Total	Percentage
1992	8	9	60	14.74	2005	19	109	207	9.65
1993	4	14	55	8.92	2006	17	127	237	7.58
1994	3	18	107	3.73	2007	30	158	340	9.11
1995	17	36	105	17.91	2008	31	190	431	7.41
1996	7	44	124	6.39	2009	29	220	511	5.86
1997	2	47	116	2.55	2010	40	261	625	6.71
1998	1	49	131	1.51	2011	45	307	666	6.90
1999	7	57	134	5.92	2012	42	350	673	6.38
2000	9	67	98	10.09	2013	47	398	733	6.67
2001	5	73	103	5.76	2014	34	433	773	4.52
2002	7	81	109	7.26	2015	27	461	766	3.91
2003	2	84	160	1.85	2016	28	490	620	4.67
2004	4	90	173	3.41	2017	16	507	578	3.28
Total							506	9091	5.66

**Table 7:** Analysis of the basic situation of each research direction.

	Paper volume	Number of citations	Percentage of citations%	Percentage of citations%	Average citation of paper	Average citations of cited papers
Sports training	160	146	90	4678	29.6	33.1
Sports biomechanics	22	17	78	603	26.6	34.0
Sports medicine	20	14	71	220	11.1	15.2
Sports physiology and biochemistry	17	15	89	149	8.7	9.8
Sports psychology	34	30	89	337	9.8	11.1
Competition rules, judging methods and laws	62	61	98	1683	26.8	27.2
Humanities and sociology of sports	106	91	86	2201	21.4	24.9
Tennis teaching	65	61	94	2179	34.4	36.7
Other	14	7	40	193	13.4	33.7
Total	507	446	88	12503	24.7	28.1

## Data Availability

The data used to support the ﬁndings of this study are available from the corresponding author upon request.
